This article has been retracted.

# Plasma D-Dimer Predicts Short-Term Poor Outcome after Acute Ischemic Stroke

**DOI:** 10.1371/journal.pone.0089756

**Published:** 2014-02-24

**Authors:** Xiao-ying Yang, Shan Gao, Jie Ding, Yan Chen, Xing-sheng Zhou, Jing-E Wang

**Affiliations:** 1 Department of Clinical Laboratory, Shanghai Jiao Tong University, Affiliated the Sixth People Hospital Fengxian Branch, Shanghai, P. R. China; 2 Department of Neurology, Shanghai Jiao Tong University, Affiliated the Sixth People Hospital Fengxian Branch, Shanghai, P. R. China; 3 Department of Neurology, Tianjin Union Medicine Center, Tianjin, P. R. China; D’or Institute of Research and Education, Brazil

## Abstract

**Objective:**

Haemostatic biomarkers associated with poor outcome in acute ischemic stroke (AIS). The objective of the study was to evaluate the predictive value of plasma D-dimer (D-D) on functional outcome at 90-day follow-up from stroke onset.

**Methods:**

We conducted a prospective, observational cohort study in the emergency department and enrolled 220 patients with AIS. Plasma D-D concentrations, determined by a particle-enhanced, immunoturbidimetric assay, were measured. Each patient’s medical record was reviewed, and demographic, clinical, laboratory and neuroimaging information was abstracted.

**Results:**

There was a positive correlation between levels of D-D and the NIHSS (r = 0.361, p<0.001), and the infarct volume (r = 0.449, p<0.001). In the 69 patients with an unfavorable functional outcome, D-D levels were higher compared with those in patients with a favorable outcome [3.24(IQR, 2.18–4.60)mg/L vs 0.88(IQR, 0.35–1.77) mg/L; p<0.001]. After adjusting for all other significant outcome predictors, D-D level remained an independent predictor for unfavorable functional outcome and mortality with an odds ratio of 2.18 (95% CI, 1.55–2.83), 3.22 (95% CI, 2.05–6.43); respectively.

**Conclusions:**

D-D levels are a useful tool to predict outcome and mortality 90-day after acute ischemic stroke and have a potential to assist clinicians.

## Introduction

Ischemic stroke is one of the major causes of death worldwide. China has 2.5 million new stroke cases each year and 7.5 million stroke survivors [1]. It places a tremendous burden on health resources in China. Timely intervention can dramatically improve outcome and reduce disability.

D-dimer(D-D), the final product of plasmin-mediated degradation of fibrin-rich thrombi, has emerged as a simple blood test that can be used in diagnostic algorithms for the exclusion of venous thromboembolism [2]. D-D levels have certain advantages over other measures of thrombin generation, because it is resistant to ex vivo activation, relatively stable, and has a long half-life [3].

It has been suggested that modestly elevated circulating D-D values reflect minor increases in bloodcoagulation, thrombin formation, and turnover of cross linked intravascular fibrin (which is partly intra-arterialin origin) and that these increases may be associated with coronary heart disease [4]. Mahé et al [5] reported that patients with higher D-D levels are at higher risk of cardiovascular events, even if they are receiving oral anticoagulants.

Goldenberg et al [6] reported that elevated D-D concentrations are prognostic of long-term neurologic outcomes in Childhood-Onset Arterial Ischemic Stroke. Elevated D-D level has also been shown to relate to early clinical progression [7], stroke subtypes [8], infarction volume [9], unfavorable outcome [10] in ischemic stroke patients and poor functional outcome after acute spontaneous intracerebral hemorrhage [11] and subarachnoid hemorrhage [12]. On the contrary, Haapaniemi et al [3] supposed that D-D levels per se are not an independent predictor for poor outcome but reflect stroke etiology. Thus, the purpose of this study was to investigate the association between plasma D-D level at admission and short-term functional outcome in Chinese patients with acute ischemic stroke (AIS).

## Subjects and Methods

### Patients and Study Design

From February 2011 to December 2012, all consecutive patients with first-ever AIS admission to the emergency department of our hospital were recruited to participate in the study. All patients were admitted within 24 hours of experiencing a new focal or global neurological event. An acute ischemic stroke was defined according to the World Health Organization criteria [13]. Brain MRI was performed routinely within 24 hours after admission. Patients were excluded if any of the following criteria were met: a delay of 24 hours from symptom recognition to admission, age younger than 18 years, coma or epileptic seizure activity, MRI could not be performed, intracranial hemorrhage, malignancy, febrile disorders, acute or chronic inflammatory disease at study enrollment. Patients who were anticoagulated before admission were also excluded.

One hundred and twenty healthy people matched for age and gender were assigned to the normal control group. Those normal cases in our study were from our hospital staff who took part in the health examination. Records of potential controls were reviewed by a neurologist (not an author) to exclude the presence of stroke, other types of diseases. The Institutional Review Committee on Human Research of Shanghai Jiao Tong University Affiliated the Sixth People Hospital Fengxian Branch approved the study protocol. All patients received oral and written information concerning the background and procedures of the study, and the patients or their relatives gave written informed consent prior to entering the study.

### Clinical Variables

At baseline, demographic data (age and sex) and history of risk factors (hypertension, diabetes mellitus, atrial fibrillation, hyperlipidemia, smoking habit and alcohol abuse) were obtained. The time from symptom recognition to admission were also recorded. At admission, the neurological deficit was quantified using the National Institutes of Health Stroke Scale (NIHSS) [14] and stroke subtype was classified according to TOAST (Trial of Org 10172 in Acute Stroke Treatment) criteria [15]. The clinical stroke syndrome was determined by applying the criteria of the Oxfordshire Community Stroke Project: total anterior circulation syndrome (TACS); partial anterior circulation syndrome (PACS); lacunar syndrome (LACS); and posterior circulation syndrome (POCS) [16]. All patients received treatment according to current guidelines. The routine treatment of patients with AIS in our institution was thrombolytic therapy, and 62 patients (28.2%) timely receive thrombolytic therapy.

### Neuroimaging

MRI with diffusion-weighted imaging (DWI) was available in all stroke patients. In patients, DWI lesion volumes were determined by one experienced neurologist unaware of the clinical and laboratory results. The infarct volume was calculated by using the formula 0.5×*a*×*b*×*c* (where *a*is the maximal longitudinal diameter, *b* is the maximal transverse diameter perpendicular to *a,* and *c* is the number of 10-mm slices containing infarct) [17].

### End Points and Follow-up

We considered the following endpoints: (1) the primary end-point was functional outcome on day 90. Functional outcome was assessed by the modified Rankin Scale (mRS, a favourable functional outcome was defined as a mRS of 0–2 points, whereas an unfavourable outcome was defined as a mRS of 3–6 points) [18]; (2) secondary end-points were all-cause mortality within 90 days. Outcome assessment was performed by one trained medical staff blinded to D-D levels with a structured interview, if discharged, with telephone interview.

### Blood Collection and Test

Blood samples of patients and controls were obtained at 7∶00 AM in the next morning of the day of admission. Blood samples were collected in 5-ml vacuum tubes containing 0.5 ml buffered sodium citrate. Plasma aliquots were collected and centrifuged at 3000 g for 10 min at ambient room temperature. Plasma was then frozen at −80 C until assayed.

D-D concentration was measured with a particle-enhanced, immunoturbidimetric assay in a calibrated SYSMEX1500 analyzer (Sysmex Corporation, Hyogo, Japan).The median level of D-D in our normal control is 0.33 mg/L, which is slightly higher than other laboratory (0.25 mg/L) [19]. The detection limit was 0.05 mg/L, and the dynamic range was from 0.05 to 30.0 mg/L. The intra-assay coefficient of variation [CV] and inter-assay CV were 1.8–37%, 2.5%–4.6%, respectively. For all measurements, levels that were not detectable were considered to have a value equal to the lower limit of detection of the assay.

### Statistical Analysis

Results are expressed as percentages for categorical variables and as medians (interquartile ranges,IQRs) for the continuous variables. Proportions were compared using the χ2 test, and the Mann–Whitney test to compare continuous variables between groups. Correlations were determined using Spearman critical value rankings. Multivariate analysis was performed by binary logistic regression analysis, which allows adjustment for confounding factors (age, the NIHSS score, infarct volume, stroke syndrome, vascular risk factors, thrombolytic therapy and other laboratory biomarkers). Results were expressed as adjusted odds ratios (OR) with the corresponding 95% confidence intervals (CIs). Receiver operating characteristic (ROC) curves were utilized to evaluate the accuracy of D-D to predict outcomes. All statistical analysis was performed with SPSS for Windows, version 19.0 (SPSS Inc., Chicago, IL, USA). Statistical significance was defined as p<0.05.

## Results

From 302 screened patients, acute ischemic stroke was diagnosed in 242 patients, and 220 completed 3- month follow-up and were included in the analysis. The median age of patients with ischemic stroke included in this study was 68 (IQR, 54–76) years and 42.3% were women. The median NIHSS score on admission was 8 points (IQR, 5–11). The median time from stroke onset to inclusion in the study was 6.2 (IQR, 3.4–13.7) hours. An unfavorable functional outcome was found in 69 patients (31.4%) with a median mRS score of 4 (IQR, 3–6). 27 patients died, thus the mortality rate was 12.3%. Basal characteristics of patients with acute ischemic stroke are provided in table 1.

**Table 1:** Basal characteristic of patients with acute ischemic stroke.

Characteristics	All	Good outcomes	Poor outcomes	p^a^
	(n = 220)	(n = 151)	(n = 69)	
Female sex (%)	42.3	41.1	44.9	NS
Age (years), median(IQR)	68(54–76)	60(51–65)	74(63–79)	<0.001
Stroke severity, median NIHSS score (IQR)	8(5–11)	3(2–6)	11(7–16)	<0.001
Infarct volume(mL, IQR)	11(7–22)	6(3–13)	18(12–59)	<0.001
Vascular risk factors no. (%)				
Diabetes mellitus	61(27.7)	30(19.9)	31(44.9)	<0.01
Hypertension	155(70.4)	95(62.9)	60(87.0)	<0.01
Hypercholesterolemia	55(25.0)	39(25.8)	16(23.2)	NS
Coronary heart disease	62(28.2)	40(26.5)	22(31.9)	NS
Atrial fibrillation	48(21.8)	32(21.2)	16(23.2)	NS
Alcohol abuse	44(20.0)	31(20.5)	13(18.8)	NS
Smoking habit	48(21.8)	32(21.2)	14(20.3)	NS
Laboratory findings (median, IQR)				
Total cholesterol (mmol L^−1^)	4.04(3.33–4.90)	4.01(3.30–4.85)	4.07(3.37–4.94)	NS
HDL (mmol L^−1^)	1.40(1.05–1.87)	1.38(1.06–1.73)	1.49(1.05–2.15)	NS
LDL (mmol L^−1^)	2.11(1.37–2.72)	2.10(1.38–2.71)	2.12(1.36–2.72)	NS
Triglycerides(mmol L^−1^)	1.30(1.05–1.63)	1.29(1.05–1.62)	1.31(1.07–1.67)	NS
Glucose(mmol L^−1^)	5.75(4.90–7.03)	5.45(4.75–6.35)	6.32(5.33–7.76)	<0.01
C-reactive protein (mgL^−1^)	4.9(3.3–8.8)	3.9 (3.0–8.1)	5.9(4.3–9.8)	<0.001
FBG(g L^−1^)	3.66(3.25–4.04)	3.17(2.87–3.69)	4.04(3.45–4.54)	<0.01
D-dimer(mg L^−1^)	1.36(0.55–3.11)	0.88(0.35–1.77)	3.24(2.18–4.62)	<0.001
Stroke syndrome no. (%)				
TACS	25(11.4)	9(6.0)	16(23.2)	<0.01
PACS	86(39.1)	59(39.1)	27(39.1)	NS
LACS	43(19.5)	28(18.5)	15(21.7)	NS
POCS	66(30.0)	55(36.4)	11(16.0)	<0.01
Stroke etiology no. (%)				
Small-vessel occlusive	37(16.8)	24(15.9)	13(18.8)	NS
Large-vessel occlusive	43(19.5)	30(19.9)	13(18.8)	NS
Cardioembolic	87(39.5)	59(39.1)	28(40.6)	NS
Other	15(6.8)	9(6.0)	6(8.7)	NS
Unknown	38(17.4)	29(19.1)	9(13.1)	NS

IQR, interquartile range; TACS, total anterior circulation syndrome; LACS, lacunar syndrome; PACS, partial anterior circulation syndrome; POCS, posterior circulation syndrome; NIHSS, National Institutes of Health Stroke Scale; HDL, High-density lipoproteins; LDL, Low-density lipoproteins;FBG, Fibrinogen.

a *p* value was assessed using Mann-Whitney *U* test or χ2 test.

Plasma D-D levels were significantly (p<0.001) higher in AIS patients as compared to normal controls [1.36 (IQR, 0.55–3.11)mg/L and 0.33 (IQR, 0.18–0.80)mg/L, respectively; Figure 1.). Interestingly, plasma D-D levels were also significantly higher in AIS patients who received thrombolytic therapy as compared to others [1.12 (IQR, 0.47–2.77)mg/L and 0.52 (IQR; 0.35–0.89)mg/L, respectively; p<0.001]. There was a positive correlation between levels of D-D and the NIHSS (r = 0.361, p<0.001; Figure 2a.) There was a modest correlation between D-D levels and age(r = 0.321, p<0.001). There was no correlation between levels of serum cortisol levels and sex (p = 0.212). In patients for whom MRI data were available (n = 220), there was a positive correlation between levels of D-D and the infarct volume (r = 0.449, p<0.001; Figure 2b.).

**Figure 1:** Plasma D-dimer levels in acute ischemic stroke patients and control group. Mann–Whitney U-test. All data are medians and in-terquartile ranges (IQR). Significantly higher in stroke patients as compared to normal cases (p<0.001).

**Figure 2:** Correlation between plasma D-dimer levels and others predictors. (a) Correlation between plasma D-dimer levels and the National Institutes of Health Stroke Scale (NIHSS) score; (b) Correlation between plasma D-dimer levels and infarct volume.

In the 69 patients with an unfavorable functional outcome, D-D levels were higher compared with those in patients with a favorable outcome [3.24(IQR, 2.18–4.60)mg/L vs 0.88(IQR, 0.35–1.77) mg/L; p<0.001). See the figure 3. With an unadjusted OR of 3.56 (95% CI, 1.99–6.34), D-D had a strong association with functional outcome. See the table 2. After adjusting for all other significant outcome predictors, D-D remained can be seen as an independent outcome predictor with an adjusted OR of 2.18 (95% CI, 1.55–2.83). See the table 2.

**Figure 3:** Plasma D-dimer levels in patients with favorable outcomes and unfavorable outcomes. Significantly higher in unfavorable patients as compared to favorable (p<0.001).

**Table 2:** Univariate and multivariate logistic regression analysis for outcome and mortality.

Parameter	Univariate Analysis			Multivariate Analysis		
	OR a	95% CI a	*P*	OR a	95% CI a	*P*
Predictor: functional outcome						
D-dimer (increase per unit)	3.56	1.99–6.34	<0.001	2.18	1.55–2.83	0.005
Age (increase per unit)	1.21	1.05–1.88	0.004	1.06	1.01–1.22	0.001
Hypertension	1.55	1.12–2.45	0.011	1.33	0.82–1.77	0.590
Diabetes mellitus	1.17	1.01–1.44	0.043	1.20	0.70–1.69	0.527
Glucose (increase per unit)	1.08	0.89–1.27	0.027	1.06	0.93–1.31	0.021
FBG(increase per unit)	1.31	1.02–1.65	0.046	1.22	0.97 –1.98	0.053
CRP (increase per unit)	1.08	0.97–1.13	0.012	1.06	1.00–1.24	0.004
Infarct volume(increase per unit)	1.16	1.10–1.22	0.003	1.11	1.01–1.29	0.006
NIHSS (increase per unit)	1.34	1.15–1.54	<0.001	1.31	1.10–1.48	<0.001
TACS	4.01	2.54–8.32	0.024	2.11	1.02–4.35	0.236
Not thrombolytic therapy	1.98	1.16–2.94	0.007	1.65	1.34–2.45	0.006
Predictor: death						
D-dimer (increase per unit)	4.25	1.93–9.28	<0.001	3.22	2.05–6.43	0.002
Age (increase per unit)	1.18	1.04–1.85	<0.001	1.06	1.03–1.09	<0.001
Hypertension	1.16	0.96–1.40	0.090	1.21	0.78–1.54	0.124
Diabetes mellitus	1.24	0.98–1.55	0.027	1.17	0.99–1.77	0.033
Glucose (increase per unit)	1.10	0.93–1.33	0.011	1.08	0.95–1.55	0.036
FBG(increase per unit)	1.40	1.05–1.78	0.033	1.42	0.95–2.07	0.027
CRP (increase per unit)	1.11	1.01–1.28	0.006	1.09	0.99–1.32	0.013
Infarct volume(increase per unit)	1.18	1.11–1.31	0.005	1.17	1.04–1.44	0.009
NIHSS (increase per unit)	1.30	1.12–1.47	<0.001	1.16	1.08–1.24	<0.001
TACS	4.87	2.14–9.02	0.036	1.55	0.56–4.63	0.423
Not thrombolytic therapy	1.96	1.20–2.86	0.005	1.62	1.11–2.87	0.006

a Note that the odds ratio corresponds to a unit increase in the explanatory variable.

OR, odds ratio; CI, confidence interval; CRP, C-reactive protein; NIHSS, National Institutes of Health Stroke Scale; TACS, total anterior circulation syndrome.

Based on the ROC curve, the optimal cut-off value of plasma D-D levels as an indicator for diagnosis of unfavorable functional outcome was projected to be 1.99 mg/L, which yielded a sensitivity of 81.2% and a specificity of 79.7%, the area under the curve was 0.84(95%CI, 0.79–0.90). See the figure 4. D-D was in the range of the NIHSS with an AUC of 0.83 (0.77–0.89) and had a higher prognostic accuracy as compared to infarct volume (AUC 0.75 (0.58–0.84), p<0.01) and C-reactive protein (AUC 0.71 (0.60–0.79), p = 0.01).

**Figure 4:** Receiver operating characteristic (ROC) curves were utilized to evaluate the accuracy of D-dimer levels to predict short-term outcomes.

D-D levels in 27 patients who died were more than 4 times greater as compared with patients who survived [3.98 (IQR, 2.25–5.69)mg/L vs 0.75(IQR, 0.32–1.48)mg/L; p<0.001). After adjustment for possible parameters, D-D level remained an independent predictor for mortality with an OR of 3.22 (95% CI, 2.05–6.43). See the table 2.

## Discussion

In this study, we firstly assessed plasma D-D levels with regard to their accuracy to predict short-term functional outcome in patients with AIS within 90 days in Chinese population. Our main finding was that elevated levels of D-D is an independent short-term prognostic marker of functional outcome and death in Chinese patients with AIS even after correcting for possible confounding factors. We also found that that plasma D-D levels increased with infarct volume and neurological deficit (assessed by the NIHSS).

These results are in accordance with the results from other studies showing that elevated levels of D-D was associated with older age, greater severity of neurological deficit, larger ischemic lesions, stroke subtypes and worse prognoses in stroke patients [8]–[9], [20]–[21]. In addition, the routine thrombolytic therapy of patients with AIS could alter D-D levels. After adjusted this condition, plasma D-D levels still can be seen as an independent prognostic marker of functional outcome and death.

Over the last two decades numerous studies have explored whether D-D measurements would help stroke clinicians. One study reported that D-D is independently related to acute stroke severity and short-term outcome [10]. Similarly,Yuan et al [7] found that D-D of acute period strongly indicates an unfavorable clinical outcome in a cohort of Chinese patients with AIS. Otherwise,Haapaniemi et al [3] suggested that regarding prediction of patient outcome, good clinical evaluation is clearly superior to D-D testing. From our results, we could confirm that plasma D-D was a valuable and independent short-term prognostic marker of functional outcome and death after stroke, and the prognostic value was in the range of clinical evaluation (assessed by the NIHSS).

Several blood biomarkers had been reported to relevant to functional outcome in AIS patients: inflammation markers [22], neuroendocrine markers [23]–[24], Vitamin D [25] and haemostatic biomarkers [20], [26]. Kang et al [26] reported that elevated levels of D-D in the 24-hour window after acute ischemic stroke are associated with early recurrence of silent brain infarcts independent of other clinical, imaging, and laboratory variables. D-D and CRP are independently associated with poor outcome in acute ischemic stroke [20]. We found that after adjusted with CRP, D-D was still associated with stroke outcome, which was in accordance with another study [27]. In addition, there was a body of evidence from other studies suggested that D-D is associated with poor outcome in acute stroke [28]–[29].

The mechanism of the hemostatic system activation and the association between D-D concentration and functional outcome in patients with AIS remains unclear. The elevation of D-D concentration thus reflects hypercoagulation and this is considered a poor prognostic factor. First, increased D-Dr levels may reflect ongoing thrombus formation within cerebral vessels or may be a marker of systemic hypercoagulability [7]. Second, D-D may stimulate the inflammatory process. Activated inflammation and activated coagulation, in concert with each other, may contribute to the development of unfavorable outcome [30]. Furthermore, high D-D levels may be resistant to the endogenous fibrinolytic system [31]. In a word, D-D is both an acute phase reactant and a marker of turnover of cross-linked fibrin, generated by activation of coagulation and fibrinolysis; hence, it may represent the biological activation of both the inflammatory, haemostatic and fibrinolytic systems. However, we cannot be certain of the biological mechanisms behind elevated D-D levels predicting acute stroke outcome, and it is necessary to exercise caution in implying causality from epidemiological studies.

There are some limitations to our study. First, our study sample was restricted to individuals with acute ischemic stroke in the first 24 hours of symptom onset and thus is not representative of stroke patients in general. In addition, a single researcher assessed consecutive admissions to the hospital using relatively few exclusion criteria, other than those to establish the diagnosis of acute ischemic stroke also should be considered. Second, we cannot exclude the possibility that D-D levels increased after stroke onset as acute phase reactants. Third, we cannot exclude the possibility that plasma D-D increased under immobile state such as aspiration pneumonia and venous thrombosis. D-D level is very rarely elevated in healthy individuals, however, may increase in many illnesses and physiological conditions associated with thrombosis and thrombolysis [3]. These patients may have had widespread vascular disease before stroke onset and are, therefore, likely to have increased pre-event levels when compared with population controls. Forth, without serial measurement of the circulating D-D levels, this study yielded no data regarding when and how long D-D is elevated in these patients. Haapaniemi et al [3] reported that following AIS, D-D levels gradually increase peaking around 2 weeks, remain high for several weeks, and then gradually decrease. Fifth, long-term MRI and clinical follow-up data were not included in the study protocol, so these relationships were not examined beyond the 90-day clinical outcome. Lastly, all patients in our study were submitted to MRI in order to obtain the MRI results. In this process, the inclusion criterion may have introduced a selection bias, where only the least severe patients (who could stand a MRI) were studied.

## Conclusions

Our study suggests that D-D levels are a useful tool to predict outcome and mortality 90-day after acute ischemic stroke in Chinese population and have a potential to assist clinicians.

## References

[1] LiuL, WangD, WongKSL, WangY (2011) Stroke and Stroke Care in China Huge Burden, Significant Workload, and a National Priority. Stroke 42: 3651–3654.2205251010.1161/STROKEAHA.111.635755

[2] Meng R, Wang X, Hussain M, Dornbos D 3rd, Meng L, et al. (2013) Evaluation of plasma d-dimer plus fibrinogen in predicting acute CVST. International Journal of Stroke, doi: 10.1111/ijs.12034. [Epub ahead of print].10.1111/ijs.12034PMC414499623506130

[3] HaapaniemiE, TatlisumakT (2009) Is D-dimer helpful in evaluating stroke patients? A systematic review. Acta Neurologica Scandinavica 119: 141–150.1870567710.1111/j.1600-0404.2008.01081.x

[4] LoweGD, RumleyA (1999) Use of fibrinogen and fibrin D-dimer in prediction of arterial thrombotic events. Thromb Haemost 82: 667–672.10605766

[5] MahéI, BergmannJF, ChassanyO, dit-SollierCB, SimoneauG, et al (2012) A multicentric prospective study in usual care: D-dimer and cardiovascular events in patients with atrial fibrillation. Thromb Res 129: 693–699.2191730210.1016/j.thromres.2011.08.014

[6] GoldenbergNA, JenkinsS, JackJ, Armstrong-WellsJ, FentonLZ, et al (2013) Arteriopathy, D-Dimer, and Risk of Poor Neurologic Outcome in Childhood-Onset Arterial Ischemic Stroke. J Pediatr 162: 1041–1046.2326010210.1016/j.jpeds.2012.11.035PMC4115645

[7] Yuan W, Shi ZH (2013) The relationship between plasma D-dimer levels and outcome of Chinese acute ischemic stroke patients in different stroke subtypes. J Neural Transm, Doi: 10.1007/s00702-013-1113-y [Epub ahead of print].10.1007/s00702-013-1113-y24201836

[8] Koch HJ, HornM, BogdahnU, IckensteinGW (2005) The relationship between plasma D-dimer concentrations and acute ischemic stroke subtypes. J Stroke Cerebrovasc Dis 14: 75–79.1790400410.1016/j.jstrokecerebrovasdis.2004.12.002

[9] ParkYW, KohEJ, ChoiHY (2011) Correlation between serum D-dimer level and volume in acute ischemic stroke. J Korean Neurosurg Soc 50: 89–94.2205322510.3340/jkns.2011.50.2.89PMC3206284

[10] BergeE, FriisP, SandsetP (2001) Hemostatic activation in acute ischemic stroke. Thromb Res 101: 13–21.1134220210.1016/s0049-3848(00)00380-7

[11] DelgadoP, Alvarez-SabinJ, AbilleiraS, SantamarinaE, PurroyF, et al (2006) Plasma D-dimer predicts poor outcome after acute intracerebral hemorrhage. Neurology 67: 94–98.1683208410.1212/01.wnl.0000223349.97278.e0

[12] JuvelaS, SiironenJ (2006) D-dimer as an independent predictor for poor outcome afteraneurysmal subarachnoid hemorrhage. Stroke 37: 1451–1456.1669090110.1161/01.STR.0000221710.55467.33

[13] HatanoS (1976) Experience from a multicentre stroke register: a preliminary report. Bull World Health Organ 54: 541–553.1088404PMC2366492

[14] BrottT, AdamsHPJr, OlingerCP, MarlerJR, BarsanWG, et al (1989) Measurements of acute cerebral infarction: A clinical examination scale. Stroke 20: 864–70.274984610.1161/01.str.20.7.864

[15] AdamsHP, BendixenBH, KappelleLJ, BillerJ, LoveBB, et al (1993) Classification of subtype of acute ischemic stroke. Definitions for use in a multicenter clinical trial. TOAST. Trial of Org 10172 in Acute Stroke Treatment. Stroke 24: 35–41.767818410.1161/01.str.24.1.35

[16] BamfordJ, SandercockP, DennisM, BurnJ, WarlowC (1991) Classification and natural history of clinically identifiable subtypes of cerebral infarction. Lancet 337: 1521–1526.167537810.1016/0140-6736(91)93206-o

[17] SimsJR, GharaiLR, SchaeferPW, VangelM, RosenthalES (2009) ABC/2 for rapid clinical estimate of infarct, perfusion, and mismatch volumes. Neurology 72: 2104–2110.1952851710.1212/WNL.0b013e3181aa5329PMC2697964

[18] BonitaR, BeagleholeR (1988) Recovery of motor function after stroke. Stroke 19: 1497–1500.320150810.1161/01.str.19.12.1497

[19] ChiuCC, LiYN, LinLJ, HsiaoCT, HsiaoKY, et al (2012) Serum D-dimer as a predictor of mortality in patients with acute spontaneous intracerebral hemorrhage. J Clin Neurosci 19: 810–813.2237763810.1016/j.jocn.2011.08.032

[20] WelshP, BarberM, LanghorneP, RumleyA, LoweGD, et al (2009) Associations of inflammatory and haemostatic biomarkers with poor outcome in acute ischaemic stroke. Cerebrovascular Dis 27: 247–253.10.1159/00019682319176958

[21] BarberM, LanghorneP, RumleyA, LoweGD, StottDJ (2006) D-dimer predictsearly clinical progression in ischemic stroke: confirmation using routineclinical assays. Stroke 37: 1113–1115.1652799810.1161/01.STR.0000209240.63821.1a

[22] WhiteleyW, JacksonC, LewisS, LoweG, RumleyA, et al (2009) Inflammatory markers and poor outcome after stroke: a prospective cohort study and systematic review of interleukin-6. PLoS medicine 6: e1000145.1990197310.1371/journal.pmed.1000145PMC2730573

[23] TuWJ, DongX, ZhaoSJ, YangDG, ChenH (2013) Prognostic value of plasma neuroendocrine biomarkers in patients with acute ischemic stroke. J Neuroendocrinol 25: 771–778.2370163810.1111/jne.12052

[24] KatanM, FluriF, MorgenthalerNG, SchuetzP, ZweifelC, et al (2009) Copeptin: a novel, independent prognostic marker in patients with ischemic stroke. Ann Neurol 66: 799–808.2003550610.1002/ana.21783

[25] TuWJ, ZhaoSJ, XuDJ, ChenH (2014) Serum 25-hydroxyvitamin D predicts the short-term outcomes of Chinese patients with acute ischaemic stroke. Clinical Science 126: 339–346.2402039510.1042/CS20130284

[26] KangDW, YooSH, ChunS, KwonKY, KwonSU, et al (2009) Inflammatory and hemostatic biomarkers associated with early recurrent ischemic lesions in acute ischemic stroke. Stroke 40: 1653–1658.1926504510.1161/STROKEAHA.108.539429

[27] BarberM, LanghorneP, RumleyA, LoweGD, StottDJ (2004) Hemostaticfunction and progressing ischemic stroke: D-dimer predicts early clinical progression. Stroke 35: 1421–1425.1507338310.1161/01.STR.0000126890.63512.41

[28] Di NapoliM, PapaF, VillaPini (2002) Stroke DataBank Investigators: Inflammation, hemostaticmarkers, and antithrombotic agents inrelation to long-term risk of new cardiovascularevents in first ever ischemic stroke patients. Stroke 33: 1763–1771.1210534910.1161/01.str.0000019124.54361.08

[29] AgenoW, FinazziS, SteidlL, BiottiMG, MeraV, et al (2002) Plasmameasurement of D -dimer levels for the earlydiagnosis of ischemic stroke subtypes. Arch Intern Med 162: 2589–2593.1245623110.1001/archinte.162.22.2589

[30] CsalaM, LérántI, BánhegyiG, KardonT, PuskásF, et al (1998) Prostaglandin-independent stimulation ofinterleukin-6 production by fibrinogen degradation product D in perfusedmurine liver. Scand J Immunol 48: 269–271.974321110.1046/j.1365-3083.1998.00395.x

[31] UrbachH, HartmannA, PohlC, OmranH, WilhelmK, et al (2002) Local intra-arterial thrombolysis in the carotid territory: does recanalization depend on the thromboembolus type? Neuroradiology 44: 695–699.1218554810.1007/s00234-002-0762-6

